# Cost-Effectiveness Analysis of Standardized Clinical Nutrition Diagnosis and Treatment Pathway in Patients with Pulmonary Infection

**DOI:** 10.1155/2022/6706390

**Published:** 2022-07-26

**Authors:** Yingyi Chen, Wenqian Zhang, Qian You, Jie Zheng, Wen Hu, Zhiyong Rao

**Affiliations:** Department of Clinical Nutrition, West China Hospital of Sichuan University, Chengdu, 610041 Sichuan, China

## Abstract

**Objective:**

From the perspective of economics, this study discusses the value of establishing a standardized clinical nutrition diagnosis and treatment pathway in the diagnosis and treatment of pulmonary infection and provides a reference for optimizing the diagnosis and treatment pathway of pulmonary infection.

**Methods:**

The patients who received the nutrition diagnosis and treatment pathway intervention in 2017 were counted as the routine group and were subdivided into the conventional intervention group (C1) and conventional control group (C2) according to whether the standardized nutrition therapy was applied or not. The patients who received the nutrition diagnosis and treatment pathway intervention in 2020 were counted as the experimental group and were subdivided into the experimental intervention group (T1) and the experimental control group (T2) according to whether standardized intervention was applied or not. The total hospitalization expenses, average daily hospitalization cost, nutrition support expenses, plasma albumin before and after nutrition support, readmission, and other indicators of all patients were recorded and compared. The cost-effectiveness ratio (CER), incremental cost-effectiveness ratio (ICER), and cost-effectiveness threshold for cost-effectiveness analysis were adopted.

**Results:**

Compared with the C2 group, the C1 group had higher total hospitalization expenses, average daily hospitalization expenses, nutritional support expenses, and plasma albumin improvement rate and lower readmission rate (*P* < 0.001). Compared with the T2 group, the T1 group had higher total hospitalization cost, average daily hospitalization expenses, nutritional support expenses, and plasma albumin improvement rate and lower readmission rate (*P* < 0.001). Taking the improvement rate of plasma albumin as the effect index, compared with the C1 group, the T1 group has less investment cost and better effect, and the ICER is negative (below the cost-effect threshold). And taking the readmission rate as the effective index, compared with the C1 group, the T1 group invested less cost and had a better effect, and the ICER was negative (below the cost-effect threshold).

**Conclusion:**

For the patients with pulmonary infection, whether the improvement rate of plasma albumin or the readmission rate is used as the impact index, the standardized nutrition diagnosis and treatment pathway in 2020 is more economical than the nonstandardized nutrition diagnosis and treatment pathway.

## 1. Introduction

Disease-associated malnutrition (disease-related malnutrition, DRM) refers to malnutrition caused by feeding and metabolic changes because of the disease [1]. The problem of increasing health costs is the main motivation for almost all government health reforms, and reasonable clinical treatment is also an important way to reduce medical costs. However, what is easily overlooked in clinical treatment is the economic burden of DRM, and the possibility of managing DRM through medical nutrition optimization is often not taken into account [2]. Patients with nutritional risk or malnutrition have worse clinical outcomes than those with no nutritional risk or malnutrition, and they can lead to high hospitalization costs, increased unplanned readmission rates, increased incidence of infectious complications, and decreased quality of life [3, 4]. However, the reason for the adverse clinical outcome may be that there is no reasonable nutrition diagnosis and treatment path. Reasonable clinical nutrition treatment is an important way to reduce medical expenses and establish a standardized clinical nutrition diagnosis and treatment pathway [5], which is the key to achieving reasonable nutritional support treatment, in addition to improving the nutritional status of patients and clinical outcome, even when the treatment effect is the same, can save medical costs for patients and even the country, which is the goal of the development of clinical nutritional treatment discipline [6, 7].

Pulmonary infection is a reaction caused by lung damage caused by viruses, bacteria, or physical and chemical factors in the lungs of patients. Most patients are in a state of high decomposition and high metabolism and often develop malnutrition. Patients with respiratory diseases can experience prolonged hospitalization, prolonged ventilator use, aggravated myasthenia gravis, increased infection, increased hospitalization cost, poor treatment effects, and so on [8]. The early detection of patients with nutritional risk and malnutrition and timely nutritional intervention are critical for disease recovery [9]. Routine nutritional support is the perioperative nutritional support program chosen by most inpatients. Although the cost is low, some patients have small benefits. After the implementation of the standardized clinical nutrition diagnosis and treatment pathway in 2020, most patients can achieve good results, but some patients are concerned that the cost of this intervention is too high. Therefore, economic evaluation of different intervention programs can provide a reference for patients to choose appropriate intervention programs.

The essence of health economic evaluation is to compare the “cost-effectiveness analysis (CEA)” of different health intervention programs. The purpose of CEA is to analyze the treatment program with the lowest cost when seeking a certain treatment. In clinical treatment, the most expensive program is not necessarily the best, and the low-cost program is not necessarily the best. Therefore, it is necessary to evaluate the ratio of the cost of an intervention program to its possible effect through CEA. The results of CEA are expressed as “cost-effectiveness ratio (CER)” and “incremental cost-effectiveness ratio (ICER).” CER directly links healthcare costs to clinical outcomes. The lower the CER, that is, the lower the input cost, the better the effect. Although CER can directly compare the resource utilization efficiency of different programs, it cannot fully reflect the cost to be paid and the health output obtained, nor the pursuit of better health outcomes. ICER represents the “difference in average cost” of the different options divided by the “difference in average effect.” The smaller the ICER value, the less the cost per unit of health outcome gained, and the more likely the option is to be economical. At the same time, the concept of threshold is also introduced in ICER's judgment; that is, considering the level of social willingness to pay for health output, it has richer decision-making information. The cost-effectiveness threshold refers to the level of cost and effectiveness that an intervention should achieve in a given health care system to be acceptable. And the ICER indicator for decision support must also specify a judgment threshold to judge which one is better than the increased health output and the increased cost [10].

Although the safety and efficacy of the main technologies for the treatment of diseases vary, the medical resources of any country are limited, and it is very meaningful to increase the economic evaluation for clinicians to choose the treatment of patients. Currently, pharmacoeconomic evaluation research is currently quite successful, but there are few economic evaluations related to medical nutrition therapy, which have problems such as a single existing evaluation index and a relatively immature evaluation method system. It is necessary to select appropriate nutrition intervention projects and adopt more targeted intervention tools and economic evaluation methods according to the actual domestic situation [11]. Our study retrospectively collected 100 pulmonary infection patients who underwent nutritional support at West China Hospital of Sichuan University in 2017 and collected 100 pulmonary infection patients who underwent nutritional support at the same hospital in 2020. In this study, based on CER and ICER, the value of different clinical nutrition diagnosis methods was compared from an economic point of view, in order to provide a reference for patients to reasonably choose intervention programs, rationally allocate health resources, and promote the development of clinical nutrition.

## 2. Data and Methods

### 2.1. Basic Information of the Participants

We retrospectively collected 100 pulmonary infection patients who underwent nutritional support at West China Hospital of Sichuan University in 2017 and collected 100 pulmonary infection patients who underwent nutritional support at the same hospital in 2020. This study was approved by the Ethics Committee of West China Hospital of Sichuan University; all patients were informed and consented.

The inclusion criteria were as follows: (1) patients admitted to West China Hospital of Sichuan University, aged 18 to 90 years old; (2) lung infection patients; and (3) patients with nutritional support after consultation.

Exclusion criteria were as follows: (1) patients under the age of 18 or over 90, (2) patients undergoing daytime surgery or staying in the hospital overnight and patients undergoing surgery before 8 o'clock the next day, (3) patients with advanced malignant tumors, (4) end-stage patients such as brain death, (5) patients with severe liver and renal function, and (6) participating in other nutritional interventions.

The grouping standard is as follows: before the implementation of the standardized clinical nutrition diagnosis and treatment pathway in 2017, the patients receiving nutritional support were in the routine group. Then, the patients were divided into a conventional intervention (C1) group and a conventional control (C2) group according to whether they received standardized nutritional treatment. The C1 group was the nutritional intervention group treated with standardized nutrition therapy, and the C2 group was the nutrition intervention group after the doctor directly consulted without a standardized nutrition treatment process. Patients after the implementation of the standardized clinical nutrition diagnosis and treatment pathway in 2020 were used as the trial group. Moreover, they were divided into the trial intervention (T1) group and trial control (T2) group according to whether they received standardized nutritional treatment. The T1 group was the nutritional intervention group treated with standardized nutrition therapy, and the T2 group was the nutrition intervention group after the doctor directly consulted without a standardized nutrition treatment process.

### 2.2. Standardized Clinical Nutrition Diagnosis and Treatment Pathway

Conventional nutrition support pathways include a single nutritional risk screening, physician assessment of nutritional status, and clinical dietitian development of nutrition treatment plans in a scattered form, without a unified pathway. The standardized clinical nutrition diagnosis and treatment pathway referred to the nutritional risk screening-nutritional status evaluation-nutrition support (intervention) action plan. Specifically, nutritional risk screening was routinely performed by the ward head nurse with an NRS 2002 nutritional risk screening scale within 24 h of admission, Grade < 3 points for patients a week after rescreening, Grade ≥ 3 points of patient HIS system for risk warning, and nutrition status evaluated by a clinical dietitian, and nutritional diagnosis was performed based on the evaluation results. Moreover, we consulted with the physician in charge to formulate an individualized nutrition intervention plan that included enteral nutritional therapy and parenteral nutrition therapy. Then, the implementation was assisted by a competent nurse, joint monitoring, and effect evaluation [12].

### 2.3. Nutrition Support Program

According to the guidelines of their Chinese Society for Parenteral and Enteral Nutrition, standardized nutritional support was defined as 25 kcal/kg/d-30 kcal/kg/d, nonprotein energy (as carbohydrate and fat), and 0.93 g/kg/d-1.25 g/kg/d protein for patients.

### 2.4. Judgment Criteria for Undernutrition

According to the reference range of the WS/T404 common clinical biochemical test project of the health industry standard of China, the normal range of albumin was 40-55 g/L, so albumin < 40 g/L was judged as malnutrition.

### 2.5. Health Economic Evaluation

The most important health economic analysis method used in this study was the cost-effectiveness ratio (CER), which directly linked medical costs to clinical treatment effects. The lower the input cost is, the better the effect. Although it could straightforwardly compare the resource use efficiency of different programs, it could not fully reflect the cost to be paid and the health output obtained, nor can it reflect the pursuit of better health effects.

Incremental cost-effectiveness ratio evaluation is the incremental input cost of marginal health improvement, which reflects the pursuit of better health output and the consideration of resource utilization efficiency. At the same time, the threshold is also introduced in the ICER judgment, which includes the consideration of the social payment willingness level of health output, with richer decision-making information. The cost-effectiveness threshold refers to the level of cost and effect that an intervention should achieve if it can be accepted under a given health care system. Also, the ICER indicator for decision support must also specify a judgment threshold to judge which is better than the increased health output and the increased cost [13].

CER and ICER were used in this study, which were used to analyze the problem from the perspective of the patient. Considering the difference in the number of hospitalization days, the cost adopted the total hospitalization cost and average (daily) hospitalization cost, and the effect was the improvement rate of plasma albumin and nonreadmission. The ICER was used for each increase in hospitalization cost, improvement in plasma albumin, and reduction in readmission rate.

The main formula is as follows:

- CER = cost (*C*)/effects (*E*)
- ICER = ∆*C*/∆*E* = increased cost/per increased unit effect

According to the evaluation conclusions of the “Guidelines for Chinese Pharmacoeconomic Evaluation Research,” if the ICER is less than or equal to the threshold, the intervention plan is more economical than the control plan. If the ICER is greater than the threshold, the result is the opposite. The threshold is recommended to be 1 to 3 times the national per gross domestic product [14]. Onefold was selected in this study.

### 2.6. Statistical Analysis

For the information and data obtained, SPSS 20.0 statistical software was selected for this analysis, and the nonparametric Wilcoxon signed rank-sum test and the *χ*^2^ test were used for data analysis. *P* < 0.05 indicated that the difference was statistically significant.

## 3. Results

### 3.1. Analysis of Hospitalization Expenses

The total hospitalization expenses, average (daily) hospitalization expenses, and nutritional support expenses were collected, and the Wilcoxon signed rank-sum test was performed for each pair of groups.

#### 3.1.1. Total Hospitalization Expenses

The total cost of hospitalization was compared between the T1 group and T2 group, *Z* = −5.936 (*P* < 0.001) and compared with the C1 group and C2 group, *Z* = −6.391 (*P* < 0.001), and the difference was statistically significant. However, the costs of the T1 group were higher than those of the T2 group; the C1 group was higher than the C2 group. The T1 group was compared with the C1 group, *Z* = −1.868 (*P* > 0.05). Although the T1 group was lower than the C1 group in terms of cost, the difference was not statistically significant (see Table 1 for details).

#### 3.1.2. Average (Daily) Hospitalization Expenses

Due to the difference in the number of hospitalization days, comparing the average (daily) hospitalization expenses, the T1 group was compared with the T2 group, *Z* = −5.887 (*P* < 0.001), and the C1 group was compared with the C2 group, *Z* = −4.833 (*P* < 0.001), The difference is statistically significant, but the cost of the T1 group was higher than that of the T2 group, and the C1 group was higher than the C2 group. Compared with the C1 group, the T1 group was lower in cost, *Z* = −1.820 (*P* > 0.05), but the difference was not statistically significant, as shown in the details in Table 2.

#### 3.1.3. Nutritional Support Expenses

Both the comparative total hospitalization cost and average (daily) hospitalization expenses were significantly higher in the intervention group than in the control group.

The cost of extracting nutritional support is compared again. The T1 group was compared with the T2 group, *Z* = −5.515 (*P* < 0.001), and the C1 group was compared with the C2 group, *Z* = −5.667 (*P* < 0.001); the difference was statistically significant. The cost of the T1 group was higher than that of the T2 group, and the C1 group was higher than the C2 group. Compared with the C1 group, the T1 group was lower, *Z* = −1.096 (*P* > 0.05), and the proportion of nutritional support expenses was higher (the cost of nutritional support in the T1 group accounted for 3.20%; the C1 group nutritional support costs accounted for 2.71%), but the difference was not statistically significant (see Table 3 for details).

### 3.2. Economic Analysis: Cost-Effectiveness Ratio and Incremental Cost-Effectiveness Ratio

First, the chi-square test was performed on the readmission rate of the four groups of inpatients, and it was found that the difference in the readmission rate of the four groups of inpatients was statistically significant (*P* < 0.05). The difference between the T1 group and the T2 group was also statistically significant (*P* < 0.05); the difference between the C1 group and the C2 group was not statistically significant (*P* > 0.05) (see Table 4 for details). There was no statistically significant difference between the T1 group and the C1 group (*χ*^2^ = 3.053, *P* = 0.081). This shows that nutrition support treatment under the “standardized clinical nutrition diagnosis and treatment pathway” can effectively reduce the readmission rate.

Taking the total hospitalization expenses and average (daily) hospitalization expenses of each group of patients as the cost and taking the percentage of improvement in plasma albumin before and after nutritional support and the rate of nonreadmission for each group as the effect, the cost-effectiveness ratio and incremental cost-effectiveness ratio were calculated according to the formula. The discount rate recommended by my country's pharmaceutical economics was used for the cost of different years, and it was generally 3% to 5% in my country. The World Health Organization recommends a cost–benefit discount rate of 3%. Comprehensively, the cost and effect of this article were both at a discount rate of 3% [15].

#### 3.2.1. Total Hospitalization Expenses

If the improvement rate of plasma albumin was used as an effect indicator, from the perspective of the cost-effectiveness ratio, the T1 group costs more than the T2 group, and the C1 group costs more than the C2 group, but the effect was better. Moreover, when the T1 group costs less than the C1 group, the effect is better, but the effect of the T1 group is higher than that of the T2 group, and the effect of the C1 group is higher than that of the C2 group. From the perspective of the incremental cost-effectiveness ratio, for every one percentage point improvement in plasma albumin, the T1 group needed an additional investment of RMB 179,800, and the C1 group needed an additional investment of RMB 262,100. Compared with the C1 group, the T1 group invested less cost and obtained better results, and the ICER was a negative value. That is, it was an advantageous plan to follow a standardized clinical nutrition diagnosis, and the treatment pathway was the superior plan.

If the rate of nonreadmission was the effect index, from the perspective of the cost-effectiveness ratio, the T1 group and C1 group cost more than the T2 group and C2 group, but the effect was higher. The T1 group was less costly than the C1 group, and the effect was better. From the perspective of the incremental cost-effectiveness ratio, to reduce the readmission rate by one percentage point, the T1 group required an additional investment of RMB 111,300, and the C1 group required an additional investment of RMB 786,400. However, the effect of the T1 group was higher than that of the T2 group, and the effect of the C1 group was higher than that of the C2 group. Compared with the C1 group, the T1 group had a negative ICER value (see Table 5 for details). This meant that it was an advantageous plan to follow the standardized clinical nutrition diagnosis and treatment pathway.

#### 3.2.2. Average (Daily) Hospitalization Expenses

Due to the large difference in the number of days of hospitalization, the economic analysis was reanalyzed based on the average daily cost. If the improvement rate of plasma albumin was used as an effect indicator, from the perspective of the cost-effectiveness ratio, the T1 group costs more than the T2 group, and the C1 group costs more than the C2 group, but the effect was better. Moreover, when the T1 group costs less than the C1 group, the effect was better. From the perspective of the incremental cost-effectiveness ratio, for every one percentage point improvement in plasma albumin, the T1 group needed an additional investment of RMB70, and the C1 group needed an additional investment of RMB80, but the effect of the T1 group was higher than that of the T2 group, and the effect of the C1 group was higher than that of the C2 group. Compared with the C1 group, the T1 group invested less cost and obtained better results, and the ICER was a negative value. That is, it was an advantageous plan to follow a standardized clinical nutrition diagnosis, and the treatment pathway was the superior plan.

If the rate of nonreadmission was the effect index, from the perspective of the cost-effectiveness ratio, the T1 group and C1 group cost more than the T2 group and C2 group, but the effect was higher. The T1 group was less costly than the C1 group, and the effect was better. From the perspective of the incremental cost-effectiveness ratio, to reduce the readmission rate by one percentage point, the T1 group required an additional investment of RMB50, and the C1 group required an additional investment of RMB23, but the effect of the T1 group was higher than that of the T2 group, and the effect of the C1 group was higher than that of the C2 group. Compared with the C1 group, the T1 group had a negative ICER value (see Table 6 for details). This means that it was an advantageous plan to follow the standardized clinical nutrition diagnosis and treatment pathway.

#### 3.2.3. Nutritional Support Expenses

If the improvement rate of plasma albumin was used as an effect indicator, from the perspective of the cost-effectiveness ratio, the T1 group costs more than the T2 group, and the C1 group costs more than the C2 group, but the effect was better. Moreover, when the T1 group costs less than the C1 group, the effect was better. From the perspective of the incremental cost-effectiveness ratio, the T1 group needed an additional investment of RMB3, and the C1 group needed an additional investment of RMB3, but the effect of the T1 group was higher than that of the T2 group, and the effect of the C1 group was higher than that of the C2 group. Compared with the C1 group, the T1 group invested less cost and obtained better results, and the ICER was a negative value; that is, it was an advantageous plan to follow a standardized clinical nutrition diagnosis, and the treatment pathway was the superior plan.

If the rate of nonreadmission was the effect index, from the perspective of the cost-effectiveness ratio, the T1 group costs more than the T2 group, and the C1 group costs more than the C2 group, but the effect was higher. The T1 group was less costly than the C1 group, and the effect was better. From the perspective of the incremental cost-effectiveness ratio, to reduce the readmission rate by one percentage point, the T1 group required an additional investment of RMB 2, and the C1 group required an additional investment of RMB 5, but the effect of the T1 group was higher than that of the T2 group, and the effect of the C1 group was higher than that of the C2 group. Compared with the C1 group, the T1 group had a negative ICER value (see Table 7 for details). This means that it was an advantageous plan to follow the standardized clinical nutrition diagnosis and treatment pathway.

### 3.3. Cost-Effectiveness Threshold

Since both more experimental and conventional groups were used, the T1 group and C1 group were more expensive than the T2 group and C2 group. Further introduce the cost-effectiveness threshold for analysis, and take 1 times the average per capita GDP as the cost-effectiveness threshold according to the “Guidelines for the Evaluation of Chinese Pharmacoeconomics.” To reduce the interference of hospitalization days, take the average per capita GDP (daily) as a comparison and convert it to RMB according to the USD exchange rate of the year (GDP of 190 yuan/day in 2017 and 160 yuan/day in 2020). The results are as follows.

If the rate of plasma albumin improvement before and after nutritional support was an effect, the incremental cost-effect ratio of the T1 group and T2 group and the incremental cost-effect ratio of the C1group and C2 group were below the threshold, suggesting that the economy of the T1 group was better than that of the T2 group and the C1 group was better than the C2 group.

If the rate of nonreadmission is an effect, the incremental cost-effect ratio of the T1 group over the T2 group is below the threshold, suggesting that the T1 group was better than the T2 group. With the C1 group incremental cost effect greater than the threshold, the C2 group was more economical (see Table 8 for details).

## 4. Discussion

The application of standardized nutritional diagnosis and treatment pathways can change the knowledge of clinical medical staff about clinical nutrition attitudes and behavior and actively implement the correct nutritional intervention programs [16]. You can better experience the clinical nutrition diagnosis and treatment process [17]. Standardized nutritional intervention can effectively prevent or improve patients' nutritional status, improve quality of life, shorten hospital stay time, reduce medical costs, reduce the occurrence of infection and other complications, reduce the unplanned readmission rate, and effectively improve the clinical outcome of hospitalized patients [18, 19]. Implementing a rational nutritional intervention program requires the discovery of patients requiring nutritional intervention. The standardized nutritional diagnosis and treatment process can just detect patients with nutritional risk and malnutrition early and choose reasonable nutritional intervention methods to prevent and correct the malnutrition of hospitalized patients [20, 21], effectively improving the clinical outcome of hospitalized patients.

### 4.1. Analysis of Hospitalization Expenses

This study found that compared with the control group, the total hospitalization expenses and average daily hospitalization expenses of the intervention group were higher in both the conventional group and the experimental group, and the difference was statistically significant. The result shows that no standardized nutritional treatment pathway seemed to be more medical cost-saving, inconsistent with the research of Miguel Montoya et al., Bonilla-Palomas et al., and Freijer et al., which believed that an effective nutritional intervention was mostly cost-saving [18, 19, 22]. This may be compared with most studies whose subjects are patients who have not received nutritional support vs. those who have undergone nutritional support, while our research subjects are all patients who have undergone nutritional support, and the intervention group is related to patients who have received nutritional support for longer periods. Barker et al. reported higher costs in malnutrition patients than in nonmalnutrition patients, with an increase in costs ranging between 45% and 102% [13]. Schuetz et al. analyzed the total cost per capita; the cost of the nutrition support cohort was too high [23]. Since we are controversial with the published conclusions, we adopt more common methods of health economics to analyze the health economic effects in several ways.

### 4.2. Analysis of Health Economics

The chi-square test was performed on the readmission rate of the four groups of admitted patients and found that nutrition support treatment under the “standardized clinical nutrition diagnosis and treatment pathway” can effectively reduce the readmission rate.

This research first adopts cost-effectiveness analysis, considering that more information can be obtained from the incremental cost-effectiveness ratio than the cost-effectiveness ratio. To obtain better results, incremental cost-effectiveness is further adopted to judge which method is more meaningful. Considering that patients with unstandardized pathways have shorter nutritional support times, shorter hospital stays, and significantly lower total expenses, the total hospitalization expenses and the average (daily) hospitalization expenses are considered costs. Considering that nutritional support expenses account for a relatively small proportion, the cost of nutritional support was compared to the cost, and the improvement rate of patients' plasma albumin and the rate of nonreadmission were used as the effects and then analyzed.

This study found that before the implementation of standardized clinical nutrition diagnosis and treatment pathway, a clinical dietitian performed nutritional risk screening for some inpatients for nutritional support. Compared with nutrition support without nutritional screening, each patient's every one percentage point improvement in plasma albumin requires an additional investment of RMB 77.7 per day, of which there is an additional RMB 3 per day (accounting for 3.9%). To reduce the readmission rate by one percentage point for a patient, an additional RMB 233.2 is required per day, of which an additional RMB 5 per day is spent on nutrition support (accounting for 2.1%).

Similarly, after the implementation of the standardized clinical nutrition diagnosis and treatment pathway in 2020, it was found that patients who implement nutrition support through standardized nutrition diagnosis and treatment pathway, compared with patients undergoing nutrition support through direct consultation, require an additional investment of RMB 73.8 per day for each improvement in plasma albumin by one percentage point, and nutrient support costs invested RMB 3 more per day (accounting for 4.1%). Every 1% reduction in the readmission rate requires an additional investment of RMB 45.7 per day, and nutrient support costs invested RMB 2 more per day (accounting for 4.4%).

This is inconsistent with most of the studies. Herbert et al. [24] found that early enteral feeding can shorten hospital stay, reduce mortality, and reduce adverse events in patients undergoing lower gastrointestinal surgery. Studies such as Wong et al.'s have found that the nutritional support team may provide cost savings and improve clinical outcomes [25]. The reason is that most studies emphasize the importance of nutritional support, while our study is mainly on whether nutrition is supported by a standardized clinical pathway, and the economic effect is not obvious. However, it can be seen that after the implementation of the “NRASA” action plan in 2020, the proportion of nutritional support has increased.

Think deeply about this issue. Compared with the original nutritional support model, standardized nutritional therapy has improved the plasma albumin of more patients and reduced the readmission rate, but it costs more. Whether it should be selected and whether it is recognized by society need further verification. Since research evaluation is a comparison of two treatment options, usually, a treatment option may increase health output while also increasing costs. However, deciding whether to adopt this treatment option requires incremental analysis, that is, judging whether to adopt this treatment option. After the treatment plan, the cost of increasing a unit of health output is worthwhile. At this time, an external reference value *λ* (also known as the cost-effectiveness threshold) needs to be introduced [14], that is, the maximum willingness to pay for an increase of a unit of health output. If the result of the incremental analysis is less than *λ*, the treatment plan is considered acceptable. In this study, 1 times GDP is selected as *λ* [6].

If plasma albumin improvement was taken as the effective index, the ICER in the 2017 routine groups and 2020 test groups were below the cost-effect threshold we set, suggesting that the standardized nutrition support program is more economical than the doctor directly asking for nutrition support in the same year. This shows that standardized nutritional support can detect patients with malnutrition earlier and conduct a timely nutritional intervention. Although the cost is higher, the effect is better, and the price is within the acceptable range [6]. If the nonreadmission rate is the effect indicator, the ICER of the routine group in 2017 was higher than the cost-effectiveness threshold we set, suggesting that it is more economical for doctors to directly ask the nutrition department for consultation than the standardized nutrition support program in the same year. The ICER of the experimental group in 2020 was lower than the cost-effectiveness threshold we set, suggesting that it is more economical to conduct a nutritional support program through a standardized nutritional diagnosis and treatment route than to directly ask the nutrition department for consultation with the doctor in the same year. This is somewhat different from other studies. Akanni et al. use quality of life years as an indicator, and the cost-effectiveness ratio is within the cost threshold. The new plan can be used as a new health promotion strategy to improve nutrition-related results, but there are also studies that use infections. Complications are an indicator of effect, and patients with nutritional support are cost-effective compared to patients without nutritional support [26].

Comparing the implementation of nutritional therapy through the standardized nutritional diagnosis and treatment pathway in 2020 with the standardized nutritional therapy before 2017, the comparison result of the discount rate conversion shows that the cost of the standardized nutritional treatment pathway is lower and the economic effect is better. This shows that it is also a standardized nutrition therapy. After the functions of each role are improved in 2020, the division of labor in each process is clear, and multidisciplinary cooperation is involved, which is more conducive to the early start of nutrition therapy and improves the effectiveness of diagnosis and treatment. This is consistent with most studies and shows that the establishment of a standardized clinical nutrition diagnosis and treatment pathway is the key to achieving reasonable nutrition support treatment, which can improve the nutritional status of patients, improve clinical outcomes, and save medical expenses for patients and the country [6, 27].

## 5. Conclusion

In summary, although the application of a standardized diagnosis and treatment pathway for nutrition requires higher costs, it can improve the nutritional status and treatment effective of patients and has cost-effect advantages and high economic value, which is worth being recommended and applied in clinical treatment. Through the analysis of health economics, the standardized nutrition diagnosis and treatment pathway can be accepted. We hope that people's views of the standardized clinical nutrition diagnosis and treatment pathway can be changed in the future to encourage everyone to accept this path and better serve clinical practice.

## Figures and Tables

**Table 1:** Comparison of the total hospitalization costs (ten thousand yuan) among the groups.

	Number of cases	*M* (*P*_25_, *P*_75_)	Wilcoxon for a two-sample rank-sum test	
			*Z* values	*P* values
Group T1	50	9.91 (5.75, 18.16)	-5.936	*P* < 0.001
Group T2	50	3.68 (2.31, 5.27)		
Group C1	50	13.44 (8.46, 22.77)	-6.391	*P* < 0.001
Group C2	50	3.52 (2.31, 5.27)		
Group T1	50	9.91 (5.75, 18.16)	-1.868	0.062
Group C1	50	13.44 (8.46, 22.77)		

**Table 2:** Comparison of average (daily) expenses (ten thousand yuan) between the groups.

	Number of cases	*M* (*P*_25_, *P*_75_)	Wilcoxon for a two-sample rank-sum test	
			*Z* values	*P* values
Group T1	50	0.43 (0.31, 0.59)	-5.887	*P* < 0.001
Group T2	50	0.23 (0.16, 0.31)		
Group C1	50	0.53 (0.35, 0.59)	-4.833	*P* < 0.001
Group C2	50	0.26 (0.17, 0.45)		
Group T1	50	0.43 (0.31, 0.59)	-1.820	0.069
Group C1	50	0.53 (0.35, 0.59)		

**Table 3:** Comparison of nutritional support expenses (ten thousand yuan) among the groups.

	Number of cases	*M* (*P*_25_, *P*_75_)	Wilcoxon for a two-sample rank-sum test	
			*Z* values	*P* values
Group T1	50	0.24 (0.14, 0.51)	-5.515	*P* < 0.001
Group T2	50	0.07 (0.04, 0.17)		
Group C1	50	0.31 (0.04, 0.17)	-5.667	*P* < 0.001
Group C2	50	0.06 (0.04, 0.17)		
Group T1	50	0.24 (0.14, 0.51)	-1.096	0.273
Group C1	50	0.31 (0.04, 0.17)		

**Table 4:** Comparison of patients' readmission status in each group.

Groups	Nonreadmission	Readmission	*χ* ^2^	*P* values	*χ* ^2^	*P* values
Group T1	48	2	10.270	0.016	9.940	0.020
Group T2	37	13				
Group C1	43	7			1.084	0.298
Group C2	39	11				

**Table 5:** Cost-effectiveness ratio and incremental cost-effectiveness ratio of total hospitalization expenses (ten thousand yuan) between each group.

Groups	Cost	Effect (%)		CER		Incremental cost	ICER	
		Plasma albumin	Nonreadmission	Plasma albumin	Nonreadmission		Plasma albumin	Nonreadmission
T1	703.86	74	96	9.51	7.33	467.48	17.98	11.13
T2	23.64	48	54	49.24	4.38			
C1	915.46	66	86	13.875	10.64	629.15	26.21	78.64
C2	286.31	42	78	6.82	3.67			
T1	644.13	68	88	9.47	7.32	-271.33	-135.67	-135.67
C1	915.46	66	86	13.87	13.87			

**Table 6:** Cost-effectiveness ratio and incremental cost-effectiveness ratio of average (daily) hospitalization expenses (ten thousand yuan) between each group.

Groups	Cost	Effect (%)		CER		Incremental cost	ICER	
		Plasma albumin	Nonreadmission	Plasma albumin	Nonreadmission		Plasma albumin	Nonreadmission
T1	0.43	74	96	0.006	0.004	0.19	0.007	0.005
T2	0.24	48	54	0.005	0.004			
C1	0.50	66	86	0.008	0.006	0.19	0.008	0.023
C2	0.32	42	78	0.009	0.004			
T1	0.39	68	88	0.006	0.004	-0.11	-0.055	-0.055
C1	0.50	66	86	0.008	0.006			

**Table 7:** Cost-effectiveness ratio and incremental cost-effectiveness ratio of average (daily) nutritional support expenses (ten thousand yuan) between each group.

Groups	Cost	Effect (%)		CER		Incremental cost	ICER	
		Plasma albumin	Nonreadmission	Plasma albumin	Nonreadmission		Plasma albumin	Nonreadmission
T1	0.0138	74	96	0.0002	0.0001	0.009	0.0003	0.0002
T2	0.0054	48	54	0.0001	0.0000			
C1	0.0137	66	86	0.0002	0.0001	0.006	0.0003	0.0005
C2	0.0075	42	78	0.0002	0.0001			
T1	0.0138	68	88	0.0002	0.0002	-0.0001	-0.00005	-0.00005
C1	0.0137	66	86	0.0002	0.0002			

**Table 8:** Average (daily) hospitalization expenses (10,000 yuan) incremental cost-effect ratio versus cost-effectiveness threshold.

Groups	ICER (plasma albumin)	ICER (nonreadmission)	Cost-effectiveness threshold
T1-T2	0.007	0.005	0.019
C1-C2	0.008	0.023	0.016

## Data Availability

Due to institutional policy restrictions, data does not support third-party sharing.
